The article "Identification of Immune-Related Prognostic Markers in Gastric Cancer" was retracted in 2023. Reasons: unreliable results or conclusions; concerns about the data; concerns about the peer review; concerns about the citations.

# Identification of Immune-Related Prognostic Markers in Gastric Cancer

**DOI:** 10.1155/2022/7897274

**Published:** 2022-03-08

**Authors:** Yanxin He, Haiping Song, Yanfang Jiang, Wanhua Ren

**Affiliations:** ^1^Department of Gastroenterology, Provincial Hospital Affiliated to Shandong University, Jinan 266042, Shandong, China; ^2^Department of Gastroenterology, The Affiliated Qingdao Central Hospital of Qingdao University, Qingdao 266000, Shandong, China; ^3^Department of Oncology, The Affiliated Qingdao Central Hospital of Qingdao University, Qingdao 266000, Shandong, China

## Abstract

Gastric cancer (GC) is a malignant tumor with a high fatality rate. Poor prognosis is the main cause of death caused by GC. In this study, the gene expression difference between GC and the control group was analyzed. Differentially expressed genes (DEGs) related to immunity were screened for enrichment analysis. The differences in immune cell infiltration and immune function between GC and normal were identified. Cox regression analysis and survival analysis were used to determine the prognostic genes of GC in TCGA and GSE62254. The potential prognostic role of genes was further evaluated by risk score. Difference genes in GC were analyzed in TCGA. Candidate genes in TCGA and GSE62254 are analyzed, and prognostic genes are determined. The potential prognostic role of genes was further evaluated by risk score. The immune-related prognostic markers in GC were determined. FABP4, LBP, LCN1, CMA1, INHBA, ANGPTL1, ACKR1, GHR, and OGN may be used as markers for monitoring the prognosis of GC in the future.

## 1. Introduction

Gastric cancer (GC) is a malignant epithelial tumor originating from mucosal cells [1]. Early patients may occasionally experience pain in the back or upper abdomen and sternum area. As the tumor grows, patients are prone to feeling full or bloating [2]. Because the symptoms are insidious and difficult to detect early, most patients with gastric cancer are in the middle and advanced stages when they see a doctor [3]. There is still no ideal treatment. Currently, GC is still treated with chemotherapy as the best method, which can prolong overall survival (OS), and there are many adverse reactions, which are difficult to tolerate in some patients and are easy to resist during treatment [4]. Due to the high heterogeneity of gastric cancer and the diverse diseased tissues, postoperative recurrence is the main reason for the short survival time of gastric cancer. In addition, this also causes the death rate of gastric cancer to rank third among all cancer patients, and the 5-year survival rate is lower than 20% [5]. Currently, monitoring methods for the prognosis of gastric cancer are still lacking. This has become an unresolved problem in current gastric cancer research.

The article "Identification of Immune-Related Prognostic Markers in Gastric Cancer" was retracted in 2023. Reasons: unreliable results or conclusions; concerns about the data; concerns about the peer review; concerns about the citations.

The Cancer Genome Atlas (TCGA), as a project supported by America, contains clinical data, genome variants, and mRNA and miRNA expression data of human cancers [6]. With sufficient breadth and specificity, and with enough research samples, reanalysis of data in TCGA has become an effective method for screening specific markers for cancer diagnosis, treatment, and prognosis monitoring [7]. In recent years, effective diagnostic markers and therapeutic targets for different cancers have been analyzed in TCGA. Genes as regulators of phenotyping have become the focus of researchers [8, 9]. During the occurrence of gastric cancer, a variety of cell transduction mechanisms are affected, and this change will inevitably cause changes in downstream target genes, which also determines the phenotypic differences between different types of cancer or the same type of cancer [2]. ACKR1 has not reported a role in GC so far, Liu et al. [10] found that CKR1 is involved in the prognosis of cervical cancer, which further implies that ACKR1 may also have a good evaluation value for the prognosis of GC. As a growth hormone receptor, GHR can promote proliferation in gastric cells in the body [11]. Meanwhile, the detection of differential gene expression in cancer not only has strong specificity but also has a relatively simple clinical application. Therefore, screening for effective target genes may become an effective tool for monitoring or treating gastric cancer [12]. However, there is a lot of research to explore effective target genes in gastric cancer. However, the currently identified genes are too single to be sensitive and specific in identifying and diagnosing the occurrence and prognosis of gastric cancer. So far, there are still few studies on the screening of prognostic markers for gastric cancer, and the screening of a database may not have a certain degree of extensiveness. Therefore, this study used the gene expression data of gastric cancer patients in different genes in the TCGA database and GSE62254 database were analyzed, and its impact on the prognosis of GC patients was evaluated. It hopes to provide a theoretical basis for future gastric cancer research and clinical application.

## 2. Materials and Methods

### 2.1. Data Processing

In TCGA, the gene expression profiles were collected in the 32 normal and 375 gastric cancer (GC) tissue. Subsequently, the gene expression profiles were analyzed by DESeq R software package. Gene expression profiles were also collected from 300 gastric tumors of gastric cancer patients in GSE62254.

The article "Identification of Immune-Related Prognostic Markers in Gastric Cancer" was retracted in 2023. Reasons: unreliable results or conclusions; concerns about the data; concerns about the peer review; concerns about the citations.

### 2.2. Survival Analysis and Cox Regression

Kaplan–Meier (K–M) estimator was performed using the survival R package. Cox regression analysis for genes in GSE62254 dataset and TCGA dataset was performed. The risk scores of the GSE62254 dataset and the TCGA dataset are calculated using Cox regression coefficients. The patients were then divided into two groups (high-risk group and low-risk group) based on the median risk score. Use the pROC R package to calculate the AUC value of the recipient.

### 2.3. Biological Function Analysis

The Gene ontology (GO) and Kyoto Encyclopedia of Genes and Genomes (KEGG) pathway enrichment analysis of DEGs were analyzed using Enrichr R package. The immune-related biological function was evaluated using Immport database.

### 2.4. Recognition of Immune-Related Genes

The genes (immune) were obtained from Immport database. The DEGs were then screened out by intersecting the immune-related genes.

### 2.5. Immune Infiltration

The immune score of each immune cell is calculated in GC patients and normals using single-sample gene set enrichment analysis (ssGSEA). A set of marker genes was yielded from Bindea et al.'s study [13].

## 3. Results

### 3.1. Differentially Expressed Genes in GC

19,929 DEGs were collected in the TCGA data (Figure 1(a)). Using Cox regression analysis, we identified 4642 genes in TCGA (Figure 1(b)). In GSE62254, 9373 genes that significantly affect the prognosis were identified in GC patients (Figure 1(c)). The results of the intersection analysis showed that a total of 435 DEGs were related to the OS of GC patients (Figure 1(d)). These genes are considered candidate genes.

### 3.2. Biological Functions of Candidate Genes

From the enrichment analysis of candidate genes, we identified a large number of GO functions (Figure 2(a)) and KEGG signaling pathways (Figure 2(b)). A total of 357 significantly enriched biological processes (BP) include extracellular matrix organization and collagen fibril organization. For 35 cellular components, collagen-containing extracellular matrix and collagen-containing extracellular matrix were enriched. The 56 molecular functions terms were enriched, such as platelet-derived growth factor binding and insulin-like growth factor II binding. Meanwhile, the candidate genes were also enriched in 21 KEGG pathways, mainly including protein digestion and absorption, cAMP signaling pathway, ECM-receptor interaction, and PI3K-Akt signaling pathway.

### 3.3. Immune-Related Genes and Cells in GC

38 candidate genes (immune-related) were identified in Immport database (Figure 3(a)). The top 10 candidate genes (FABP4, LBP, LCN1, CMA1, OBP2B, INHBA, ANGPTL1, ACKR1, GHR, and OGN) with the largest absolute values of Cox regression coefficients in the TCGA dataset as key genes (Figure 3(b)) were selected. On the other hand, to identify the role of immune cells in GC, tumor and normal immune cell infiltration is analyzed (Figure 3(b)). Subsequently, we have identified that activated CD4 T cell, CD56dim natural killer cell, central memory CD4 T cell, natural killer T cell, regulatory T cell, and type 2 T-helper cell have increased infiltration in GC patients. Effector memory CD4 T cell, eosinophil, immature dendritic cell, macrophage, mast cell, neutrophil, and T follicular helper cell have decreased infiltration in GC patients. In addition, in the Immport database, we identified the difference between immune-related biological functions between GC and normal (Figure 3(c)). Interferon receptor, interferons, interleukins, and TNF family members were activated in GC, chemokine receptors, cytokine receptors, cytokines, TGF*β* family member receptor, and TGF*β* family member were inhibited.

The article "Identification of Immune-Related Prognostic Markers in Gastric Cancer" was retracted in 2023. Reasons: unreliable results or conclusions; concerns about the data; concerns about the peer review; concerns about the citations.

### 3.4. Key Genes of GC Affect the Prognosis

The risk scores of FABP4, LBP, LCN1, CMA1, OBP2B, INHBA, ANGPTL1, ACKR1, GHR, and OGN were evaluated and divided into two groups (high-risk group and low-risk group). In the TCGA data set, the expression of FABP4, LBP, LCN1, CMA1, INHBA, ANGPTL1, ACKR1, GHR, and OGN is classified as a high-risk group, and the expression of OBP2B is classified as low-risk group (Figure 4(a)). In GC patients, AUC values were 0.65 in predicted 1-year and 3-year survival (Figure 4(b)). Compared with a low-risk group, patients with high-risk group have a worse prognosis (Figure 4(c)). In GSE62254 dataset, FABP4, LBP, CMA1, INHBA, ANGPTL1, ACKR1, GHR, and OGN were highly expressed in the high-risk group, and LCN1 and OBP2B were upregulated in the low-risk group (Figure S1A). Median risk: the AUC value of predicted 1-year and 3-year survival of GC patients is 0.7, and the AUC value of 5-year survival is 0.68 (Figure S1B). Compared with low-risk scores, the deterioration of the prognosis increases with the increase of the high-risk score (Figure S1C).

Furthermore, we calculated the differentially infiltrated immune cells between high- and low-risk groups in the TCGA dataset (Figure 5(a)). There is a significant difference in the level of infiltration of most immune cells between the two groups. Most of the immune-related biological functions identified in the Immport database have significant differences between high- and low-risk groups (Figure 5(b)).

## 4. Discussion

In this study, 35 DEGs related to the OS of GC were screened. These DEGs are mainly enriched in protein digestion and absorption, ECM-receptor interaction, and PI3K-AKT and cAMP signaling pathways. Among them, FABP4, LBP, LCN1, CMA1, INHBA, ANGPTL1, ACKR1, GHR, and OGN have good detection values for prognostic status.

The article "Identification of Immune-Related Prognostic Markers in Gastric Cancer" was retracted in 2023. Reasons: unreliable results or conclusions; concerns about the data; concerns about the peer review; concerns about the citations.

During the occurrence of gastric cancer, a variety of cell transduction mechanisms are affected, and this change will inevitably cause changes in downstream target genes, which also determines the phenotypic differences between different types of cancer or the same type of cancer [2]. Currently, GC is still treated with chemotherapy as the best method, which can prolong overall survival (OS); there are many adverse reactions, which are difficult to tolerate in some patients and are easy to resist during treatment [4]. In addition, this change also provides us with opportunities to treat and monitor the occurrence, treatment, and prognosis of cancer. In this study, we screened 435 DEGs of GC patients in the TCGA and GSE62254. These genes are mainly enriched in protein digestion and absorption, ECM-receptor interaction, and PI3K-AKT and cAMP signaling pathways. This result is similar to previous research results [14]. This also further indicates that these DEGs are related to GC.

The immune system is the most effective defense mechanism for human diseases. In normal tissues and organs, the immune level is always in dynamic balance [15]. When the body is in the pathological process, a variety of signal pathways are affected, and through the cascade effect conduction, it will eventually cause the change of downstream genes and finally cause the change of phenotype. Cancer cells continue to proliferate rapidly due to their heterogeneity, and signal transduction must have changed [16]. The study of altered signal transduction is beneficial to us for the development, treatment, and monitoring of cancer. In previous studies, the role and changes of immunity in the progression of GC have also been demonstrated [17, 18]. In this study, we further screened prognostic-related genes and finally found that FABP4, LBP, LCN1, CMA1, INHBA, ANGPTL1, ACKR1, GHR, and OGN may be potential prognostic markers. Among them, previous reports have shown that FABP4 and CMA1 have extremely high diagnostic values for the diagnosis and prediction of GC [19, 20]. LBP has a certain anticancer effect [21]. The expression of INHBA increases with the increase of GC; when knocked down, it also significantly inhibits the process of GC, which indicates that INHBA may be involved in the occurrence of GC [22]. Although ACKR1 has not reported a role in GC so far, Liu et al. [10] found that CKR1 is involved in the prognosis of cervical cancer, which further implies that ACKR1 may also have a good evaluation value for the prognosis of GC. As a growth hormone receptor, GHR can promote proliferation in gastric cells in the body [11]. Meanwhile, in the study of Ran et al. [23], low GHR expression can reduce gastric cancer cell proliferation. As a tumor suppressor, OGN can significantly inhibit the growth of tumor cells [24]. Moreover, studies have shown that its expression in GC tissues is significantly reduced [24], and the mechanism of OGN in the progression of gastric cancer has not yet been reported. At the same time, there is no relevant research on GC on the effects of LCN1 and ANGPTL1 on GC and its mechanism. However, LCN1 and ANGPTL1 have high therapeutic and diagnostic value in other cancer research [25, 26].

The article "Identification of Immune-Related Prognostic Markers in Gastric Cancer" was retracted in 2023. Reasons: unreliable results or conclusions; concerns about the data; concerns about the peer review; concerns about the citations.

## 5. Conclusion

In this study, our results show that immune response has extremely high monitoring value for cancer prognosis. Among them, FABP4, LBP, LCN1, CMA1, INHBA, ANGPTL1, ACKR1, GHR, and OGN may be used as markers for monitoring the prognosis of GC in the future. However, there is no relevant research on GC on the effects of LCN1 and ANGPTL1 on GC and its mechanism. We still need more research to explore the mechanism of action of LCN1 and ANGPTL1. In this study, we only determined that these genes may be used as symbols for prognostic tests. In the future, we will conduct more experiments to determine the key indicators.

## Figures and Tables

**Figure 1:** Differentially expressed genes affecting the prognosis of gastric cancer patients. (a) Differentially expressed genes between gastric cancer and normal control in TCGA dataset. (b) Volcano plot of Cox regression coefficients for genes affecting prognosis of gastric cancer patients in TCGA data. (c) Volcano plot of Cox regression coefficients for genes affecting prognosis of gastric cancer patients in GSE62254 data. (d) Screening of differentially expressed genes affecting the prognosis of gastric cancer patients.

**Figure 2:** GO and KEGG pathway enrichment of candidate genes. (a) The top 10 results of biological process (BP), cellular component (CC), and molecular function (MF) of GO analysis. (b) The significantly enriched KEGG pathways of candidate genes.

**Figure 3:** Identification of key genes and immune-related functions in gastric cancer. (a) Screening of candidate genes related to immunity. (b) The top 10 genes with the highest absolute value of Cox regression coefficient were taken as the key genes, and their differential expression in GC and normal. (c) Differential infiltration of immune cells in GC and normal. (d) Differences of immune-related functions in Immport database between GC and normal.

**Figure 4:** Cox risk score of key genes influences gastric cancer patient prognosis in TCGA. (a) Distribution of candidate mRNAs‐based risk scores, mRNAs expression levels, and patient survival durations in the TCGA. (b) AUC values for the risk median score to predict 1-year and 3-year survival of GC patients. (c) Kaplan–Meier curves of OS for GC patients based on the risk score in the TCGA dataset.

The article "Identification of Immune-Related Prognostic Markers in Gastric Cancer" was retracted in 2023. Reasons: unreliable results or conclusions; concerns about the data; concerns about the peer review; concerns about the citations.

**Figure 5:** Differences in immune cells and immune functions between high- and low-risk groups in TCGA. (a) Differential infiltration of immune cells in high- and low-risk groups. (b) Differences of immune related functions in Immport database between high- and low-risk groups.

## Data Availability

The datasets used and/or analyzed during the current study are available from the corresponding author on reasonable request.

## Supplementary Materials

Supplementary Materials
*Figure S1.* Cox risk score of key genes influences gastric cancer patient prognosis in GSE62254. (A) Distribution of candidate mRNAs‐based risk scores, mRNAs expression levels, and patient survival durations in the GSE62254. (B) AUC values for the risk median score to predict 1-year, 3-year, and 5-year survival of GC patients. (C) Kaplan–Meier curves of OS for GC patients based on the risk score in the GSE62254 dataset.
